The article "LncRNA MALAT1 promotes tenogenic differentiation of tendon-derived stem cells via regulating the miR-378a-3p/MAPK1 axis" was retracted in 2026. Reasons: concerns about the data; concerns about the results or conclusions.

# LncRNA MALAT1 promotes tenogenic differentiation of tendon-derived stem cells via regulating the miR-378a-3p/MAPK1 axis

**DOI:** 10.1080/21655979.2022.2076507

**Published:** 2022-05-29

**Authors:** Zhe Zhao, Jianquan Liu, Zhiqin Deng, Xiaoqiang Chen, Wencui Li

**Affiliations:** Foot and Ankle & Hand Surgery Department, Shenzhen Second People’s Hospital, the First Affiliated Hospital of Shenzhen University, Shenzhen, Guangdong, China

**Keywords:** Tendinopathy, MALAT1, tenogenic differentiation, MAPK1

## Abstract

Tendinopathy is a type of chronic injury caused by repeated pulling. Previous studies have reported that long non-coding RNA MALAT1 (MALAT1) regulates a variety of genes affecting bone metabolism. This study aimed to explore the role of the MALAT1 in tendon injury *in vivo* and *in vitro*. Human tendon-derived stem cells (TDSCs) were treated with TGF β1. Eighteen Sprague-Dawley rats were used to establish the tendinopathy animal model. Sirius Red staining and colorimetric assays were conducted to analyze the collagen content. RT-qPCR was performed to measure the mRNA levels. Western blotting was performed to measure the MAPK1 protein levels. Additionally, hematoxylin and eosin (HE) and immunohistochemical staining were used to analyze the cell number and the content of collagen type 1 and Thbs, respectively. MALAT1 expression was upregulated in TGF β1 treated TDSCs, and MALAT1 knockdown downregulated Scleraxis, Mohawk homeobox, Collagen 1A1, Fibromodulin, Matrix metallopeptidase 3, and Thrombospondin 4 in TGF β1 treated TDSCs. Bioinformatics analysis showed that miR-378a-3p was the target of MALAT1 and MAPK1, and dual-luciferase reporter assay indicated that both MALAT1 and MAPK1 could bind to miR-378a-3p. Furthermore, miR-378a-3p knockdown reversed the effect of si-MALAT1, whereas overexpression of MAPK1 reversed the effect of the miR-378a-3p mimic. Finally, MALAT1 expression was downregulated in tendinopathy rats, and MALAT1 overexpression healed tendon injury in them. MALAT1 regulated the tenogenic differentiation of TDSCs by regulating the miR-378a-3p/MAPK1 axis. Our results therefore indicate that targeting the MALAT1/miR-378a-3p/MAPK1 axis may be a promising avenue for the treatment of tendinopathy.

## Highlights

- MALAT1 was significantly upregulated in TGFβ1-treated TDSCs.
- Knockdown of MALAT1 suppressed tenogenic differentiation.
- MALAT1 functioned as a sponge for miR-378a-3p.

## Introduction

Tendinopathy is a type of chronic injury caused by repeated pulling and is characterized by motion-related pain, increased sensitivity of the local Achilles tendon, and changes in imaging of the tendon [1]. Previously, tendinopathy was thought to be a simple inflammatory reaction, and was therefore called “tendinitis”. However, recent histopathological studies have shown that the pathological process of tendinopathy involves tendon degeneration [2], and its specific pathophysiological changes need to be clarified in detail. Local stem cells are known to promote the repair of damaged tissues [3]. In 2007, Bi et al. [4] first identified a cell type different from other mesenchymal stem cells in mouse and human tendons, named the tendon stem cell (TSC). Compared to tendon cells, TSCs exhibit better cell proliferation and collagen formation abilities. TSCs differentiate into tendon cells under certain physiological conditions, and secrete extracellular matrix (ECM) components [5,6]. The differentiation of the tendon and the formation of the tendon ECM can effectively heal tendon injury. TSCs have been reported to directly participate in the repair of damaged tendons and improvement of the biomechanical properties of diseased tendons [7]. Additionally, TSCs differentiate into adipocytes, osteocytes, and chondrocytes under certain pathological conditions. Therefore, promoting the differentiation of TSCs into tenogenic cells and inhibiting their non-tenogenic differentiation under pathological conditions is an effective strategy for the treatment of tendon injury.

The article "LncRNA MALAT1 promotes tenogenic differentiation of tendon-derived stem cells via regulating the miR-378a-3p/MAPK1 axis" was retracted in 2026. Reasons: concerns about the data; concerns about the results or conclusions.

In recent years, there have been rapid strides in research on long non-coding RNAs (lncRNAs). lncRNAs are RNA transcripts with a length of more than 200 nucleotides (nt) [8,9], and have been reported to be involved in various biological processes. Emerging evidence indicates that lncRNAs are closely associated with cell differentiation and tissue regeneration [10]. However, studies on the role of lncRNAs in tenogenic differentiation are limited. In 2003, lncRNA metastasis-associated lung adenocarcinoma transcript 1 (MALAT1) was first discovered in a study on non-small cell lung cancer (NSCLC) and has attracted attention of researchers in recent years [11]. MALAT1 is approximately 8000 nt long, and is located on chromosome 11q13 [12]. Previous studies have reported that MALAT1 regulates a variety of genes affecting bone metabolism, such as upregulation of osterix protein expression to promote osteoblast proliferation and differentiation, and downregulation of RANKL expression to inhibit osteoclast activation [13,14]. However, the mechanisms underlying the role of MALAT1 in tendinopathy are still unclear. MicroRNAs (miRNAs) are small non-coding RNAs with a length of 18–22 nt [15], and perform their biological functions by competing with lncRNAs [16]. For instance, MALAT1 promotes osteoblast growth by regulating the miR-34c/SATB2 axis [17]. Zhang et al. also found that MALAT1 participates in proliferation, apoptosis, and ECM degradation, by regulating the miR-150-5p/AKT3 axis [18]. A previous study showed that miR-378a can be used as a novel biomarker for the diagnosis of tendon injury [19].

The article "LncRNA MALAT1 promotes tenogenic differentiation of tendon-derived stem cells via regulating the miR-378a-3p/MAPK1 axis" was retracted in 2026. Reasons: concerns about the data; concerns about the results or conclusions.

Therefore, in this study, we aimed to explore the role of MALAT1 in tendinopathy both *in vivo* and *in vitro*. We hypothesized that MALAT1 promotes tenogenic differentiation by regulating the miR-378a-3p/MAPK1 axis.

## Materials and methods

### Animal experiments

Eighteen Sprague-Dawley rats (210 ± 11.2 g) were provided by the Laboratory Animal Center of the Guangdong Medical University, China. The specific grouping was as follows: control group (CON), collagenase I group (Model), and Model+MALAT1 overexpression group (oe-MALAT1). In the Model group, 2.5% pentobarbital sodium was administered to anesthetize the rats. Next, 30 μL of collagenase I was injected into the bilateral Achilles tendons of the rats. Adenoviruses containing the MALAT1 overexpression vector (RiboBio, Guangzhou, China) were injected into the model group mice via the tail vein to overexpressed the MALAT1 levels. After six weeks, the rats were euthanized and the patellar tendons were collected for further analysis.

### HE staining

Patellar tendons were fixed in 4% paraformaldehyde for 24 h [20]. The tissues were then embedded in paraffin and sectioned. After washing with PBS, the sections were stained with hematoxylin and eosin. Finally, the sections were observed under a microscope (Leica Microsystems, Germany).

### Immunohistochemistry

The sections were hydrated using different concentrations of ethanol [21]. Bovine serum albumin (1%) was used for blocking. The sections were then incubated with anti-collagen I (Abcam, UK) and anti-thrombospondin 4 (THbs4) (Abcam) overnight. On the second day, the sections were treated with donkey anti-rabbit HRP-binding secondary antibody (Abcam) for 1 h, followed by addition of 3,39-diaminobenzidine tetrahydrochloride. Finally. ImageJ software was used to measure the percentage of stained area relative to the total area under a microscope (Leica Microsystems).

### Cell culture and treatment

Human tendon-derived stem cells (TDSCs) were provided by cell bank of the Chinese Academy of Sciences (Shanghai, China). TDSCs were cultured in low-glucose DMEM (10% FBS, 100 U/ml penicillin, and 100 mg/ml streptomycin) at 37°C and 5% CO_2_. For tenogenic differentiation, TDSCs were treated with 5 ng/ml TGFβ1. When cell fusion reached 70%, the cells were collected for subsequent experiments.

### Cell transfection

siRNA targeting MALAT1 (si-MALAT1 1#, si-MALAT1 2#) and siRNA negative control (si-nc), MALAT1 overexpression plasmid (oe-MALAT1) and its empty vector (oe-nc), miR-378a-3p mimic (mimic) and its negative control (nc-mimic), miR-378a-3p inhibitor (inhibitor) and its negative control (nc-inhibitor), and MAPK1 overexpression plasmid (MALAT1) and its empty vector (vector), were purchased from GenPharma. Lipofectamine 3000 (Invitrogen) was used to transfect the TDSCs, according to the manufacturer’s instructions [22].

The article "LncRNA MALAT1 promotes tenogenic differentiation of tendon-derived stem cells via regulating the miR-378a-3p/MAPK1 axis" was retracted in 2026. Reasons: concerns about the data; concerns about the results or conclusions.

Sirius Red staining

Sirius Red staining and colorimetric assays were performed to analyze the collagen content [23]. Briefly, TDSCs were washed and fixed in 4% paraformaldehyde for 10 min. The TDSCs were then stained with 1 mL saturated picric acid solution with 0.1% Sirius Red. Subsequently, 0.1% NaOH and absolute methanol were added to elute the color. Finally, a spectrophotometer (BioTek Instruments, USA) was used to quantify the red color at 540 nm.

RT-qPCR

Total RNA from the cells and tissues was separated using TRIzol® (Thermo Fisher Scientific, MA, USA). Then, the Prime Script RT Master Mix kit (Takara, Dalian, China) was used to synthesize cDNAs. PCR was performed using a miScript SYBR Green PCR Kit (Takara) on a 7900 Real-Time PCR System (Thermo Fisher Scientific, MA, USA). The reaction conditions were as follows: 95°C, 5 s; 45 cycles of 95°C, 5 s; 60°C, 1 min; 95°C, 5 s; 60°C, 1 min. The relative expression of target genes was calculated using the 2^−ΔΔCt^ method [24]. GAPDH or U6 was used as a housekeeping gene control. The primer sequences were as follows:

MALAT1, forward primer: 5’-TCCTAAGGTCAAGAGAAGTGTCAG-3’, reverse primer: 5’-GTGGCGATGTGGCAGAGAA-3’;

Scleraxis (Scx), forward primer: 5’-CTGGCCTCCAGCTACATTTCT-3’, reverse primer: 5’-GTCACGGTCTTTGCTCAACTT-3’;

Mohawk homeobox (Mkx), forward primer: 5’-CTCGCAGATGACGCTAGTGC-3’, reverse primer: 5’-TGGCTGTCGAACGGTATTCTT-3’;

Collagen 1A1 (Col1a1), forward primer: 5’-GAGGGCCAAGACGAAGACATC-3’, reverse primer: 5’-CAGATCACGTCATCGCACAAC-3’;

Fibromodulin (Fmod), forward primer: 5’-ATTGGTGGTTCCACTACCTCC-3’, reverse primer: 5’-GGTAAGGCTCGTAGGTCTCATA-3’;

Matrix metallopeptidase 3 (Mmp3) forward primer: 5’-CGGTTCCGCCTGTCTCAAG-3’, reverse primer: 5’-CGCCAAAAGTGCCTGTCTT-3’;

Thrombospondin 4 (Thbs4), forward primer: 5’-TGCTGCCAGTCCTGACAGA-3’, reverse primer: 5’-GTTTAAGCGTCCCATCACAGTA-3’;

miR-378a-3p, forward primer: 5’-GCGCACTGGACTTGGAGTC-3’, reverse primer: 5’-GCAGGGTCCGAGGTATTC-3’;

Mitogen Activated Protein Kinase1 (MAPK1), forward primer: 5’-TGAGCCGACCCTTTCAGTC-3’, reverse primer: 5’-AGCCCAATGACGTTCTCATGC-3’;

GAPDH, forward primer: 5’-TGTGTCCGTCGTGGATCTGA-3’, reverse primer: 5’-CCTGCTTCACCACCTTCTTGA-3’;

U6, forward primer: 5’-GCTTCGGCAGCACATATACTAA-3’, reverse primer: 5’-AACGCTTCACGAATTTGCGT-3’.

The article "LncRNA MALAT1 promotes tenogenic differentiation of tendon-derived stem cells via regulating the miR-378a-3p/MAPK1 axis" was retracted in 2026. Reasons: concerns about the data; concerns about the results or conclusions.

### Bioinformatics analysis

The target miRNA of MALAT1 was predicted using online Starbase software (http://hopper.si.edu/wiki/mmti/Starbase). The target of miR-378a-3p was predicted using TargetScan software (http://www.targetscan.org/vert_72/) and MiRDB software (http://mirdb.org/index.html) [25].

### Dual-luciferase reporter assay

The wild-type (WT) and mutant (MUT) 3’-UTR regions of MALAT1 or MAPK1 were cloned into the p-GL3.0 plasmid (Promega, Madison, WI, USA) to construct dual luciferase reporter vectors. The miR-378a-3p mimic and the WT and MUT 3’-UTR regions of MALAT1 or MAPK1 were co-transfected into TDSCs. After 48 h of conventional culture, fluorescence was determined using a dual-Glo luciferase assay system (Promega, Madison, WI, USA) [26].

### Statistical analysis

Data were analyzed using SPSS (version 22.0, SPSS, Chicago, IL, USA) and expressed as mean ± standard deviation. Each experiment was repeated three times. Student’s t-test was used to analyze the differences between two groups, one-way ANOVA was used to analyze the differences among multiple groups. Statistical significance was set at p < 0.05.

## Results

### Characterization of TDSCs

TDSCs have a typical fusiform morphology and can differentiate into adipocytes, osteoblasts and chondrocytes (Figure 1(a)). As shown in Figure 1 b and C, the expression levels of positive markers CD90, CD106 and CD44 were 99.54%, 99.73% and 98.79%, respectively, and those of negative markers CD105 and CD11B were 1.18% and 2.97%, respectively.

**Figure 1.** Characterization of TDSCs. (a) Morphology of TDSCs and the potential of multilineage differentiation of TDSCs. (b) Surface markers including CD90, CD105, CD44, CD106 and CD11B measured by flow cytometry assay.

### MALAT1 was significantly upregulated in the TGFβ1 treated TDSCs

We used 5 ng/ml TGFβ1 to induce tenogenic differentiation. The results showed that TGFβ1 promotes the production of collagen, and can therefore successfully induce tenogenic differentiation in TDSCs (Figure 2(a)). We also found that MALAT1 expression was upregulated in TGFβ1 treated TDSCs on days 0, 3, 7, and 10 (Figure 2(b)), and reached its highest level on day 7; therefore, we treated TDSCs with TGFβ1 for 7 days in subsequent experiments.

**Figure 2.** MALAT1 was significantly up-regulated in the TGFβ1-treated TDSCs. (a) Sirius Red staining of TDSCs treated with TGFβ1 on day 0, 3, 7, 10. (b) RT-qPCR was conducted to measure the MALAT1 expression on day 0, 3, 7, 10. *P < 0.05, **P < 0.01, ***P < 0.001.

### Knockdown of MALAT1 suppressed tenogenic differentiation

We further explored the role of MALAT1 in tenogenic differentiation. We designed an siRNA to downregulate MALAT1 expression. MALAT1 expression was dramatically downregulated after si-MALAT1 transfection (Figure 3(a)). Furthermore, MALAT1 knockdown decreased TGFβ1 induced collagen production (Figure 39b-c)). Next, we determined the expression of tenogenic markers and found that, compared with the NC group, the expression levels of Scx, Mkx, Fmod, Col1a1, Mmp3, and Thbs4 were significantly increased. Knockdown of MALAT1 reversed these effects (Figure 3(d-i)).

The article "LncRNA MALAT1 promotes tenogenic differentiation of tendon-derived stem cells via regulating the miR-378a-3p/MAPK1 axis" was retracted in 2026. Reasons: concerns about the data; concerns about the results or conclusions.

**Figure 3.** Knockdown of MALAT1 suppressed the tenogenic differentiation. (a) Transfection efficiency of si-MALAT1. (b, c) Sirius Red staining and OD value measurement of TDSCs on day 7. **d-i** RT-qPCR was conducted to measure the expressions of SCX, Mkx, COL1a1, Fmod, Mmp3 and Thbs4. *P < 0.05, **P < 0.01, ***P < 0.001.

### MALAT1 functions as a sponge for miR-378a-3p

The binding sites of MALAT1 and miR-378a-3p were predicted using the online database Starbase 3.0 (Figure 4(a)). Dual-luciferase reporter assay showed that the miR-378a-3p mimic significantly inhibited luciferase activity in TDSCs transfected with WT-MALAT1 instead of MUT-MALAT1 (Figure 4(b)). In addition, knockdown of MALAT1 upregulated the expression of miR-378a-3p, whereas overexpression of MALAT1 downregulated the expression of miR-378a-3p (Figure 4(c)). The expression of miR-378a-3p was down-regulated in the TGFβ1 group (Figure 4(d)).

**Figure 4.** MALAT1 functioned as the sponge of miR-378a-3p. (a) Bioinformatic prediction of binding site of miR-378a-3p by MALAT1. (b) Relative luciferase activity of cells after co-transfection with wild type (WT) or mutant (Mut) lncRNA MALAT1 3’-UTR reporter genes and miR-378a-3p mimics. (c) RT-qPCR was conducted to measure the relative expression of miR-378a-3p after si-MALAT1 and oe-MALAT1 transfection. (d) RT-qPCR was conducted to measure the relative expression of miR-378a-3p in the TGFβ1-treated TDSCs. ***P < 0.001.

### Knockdown of miR-378a-3p reversed the effect of si-MALAT1

Subsequently, we designed a miR-378a-3p inhibitor to downregulate miR-378a-3p expression. The expression of miR-378-3p markedly decreased after transfection with the inhibitor (Figure 5(a)). Furthermore, we found that knockdown of miR-378a-3p reversed the effects of si-MALAT1 on collagen production (Figure 5(b-c)) and the expression of Scx, Mkx, Fmod, Col1a1, Thbs4, and Mmp3 (Figure 5(d-i)).

**Figure 5.** Knockdown of miR-378a-3p reversed the effect of si-MALAT1. (a) Transfection efficiency of si-MALAT1 miR-378a-3p inhibitor. (b, c) Sirius Red staining and OD value measurement of TDSCs on day 7 after si-MALAT1 and miR-378a-3p inhibitor transfection. (d-i) RT-qPCR was conducted to measure the expressions of SCX, Mkx, COL1a1, Fmod, Mmp3 and Thbs4 after si-MALAT1 and miR-378a-3p inhibitor transfection. *P < 0.05, **P < 0.01, ***P < 0.001.

The article "LncRNA MALAT1 promotes tenogenic differentiation of tendon-derived stem cells via regulating the miR-378a-3p/MAPK1 axis" was retracted in 2026. Reasons: concerns about the data; concerns about the results or conclusions.

### Interaction between miR-378a-3p and MAPK1

The target genes of miR-378a-3p were predicted using miRDB and TargetScan. The binding sites of MAPK1 and miR-378a-3p are shown in Figure 6(a). Dual-luciferase reporter assay showed that the miR-378a-3p mimic significantly inhibited luciferase activity in TDSCs transfected with WT-MAPK1 instead of MUT-MAPK1 (Figure 6(b)). Knockdown of miR-378a-3p upregulated the expression of MAPK1 and overexpression of miR-378a-3p downregulated the expression of MAPK1 at mRNA and protein levels (Figure 6(c-d)). In addition, the expression of MAPK1 was upregulated in the TGFβ1 group (Figure 6(e)).

**Figure 6.** Interaction between miR-378a-3p and MAPK1. (a) Bioinformatic prediction of binding site of miR-378a-3p by MAPK1. (b) Relative luciferase activity of cells after co-transfection with wild type (WT) or mutant (Mut) MAPK1 3’-UTR reporter genes and miR-378a-3p mimics. RT-qPCR (c) and western blot (d) was conducted to measure the relative expression of MAPK1 after miR-378a-3p mimic and inhibitor transfection. (eS) RT-qPCR was conducted to measure the relative expression of MAPK1 in the TGFβ1-treated TDSCs. ***P < 0.001.

### Overexpression of MAPK1 reversed the effect of miR-378a-3p mimic

MAPK1 expression was significantly upregulated at both mRNA and protein levels after transfection of MAPK1 in TDSCs (Figure 7(a-b)). Overexpression of miR-378a-3p decreased collagen production, and MAPK1 suppressed the effect of the miR-378a-3p mimic (Figure 7(c-d)). In addition, compared with the TGFβ1 group, the expression levels of Scx, Mkx, Fmod, Col1a1, Mmp3 and Thbs4 decreased after transfection with the miR-378a-3p mimic. The overexpression of MAPK1 exhibited the opposite effect (Figure 7(e-j)).

**Figure 7.** Overexpression of MAPK1 reversed the effect of miR-378a-3p mimic. (a-b) Transfection efficiency of MAPK1 vector. (c-d) Sirius Red staining and OD value measurement of TDSCs on day 7 after miR-378a-3p mimic and MAPK1 vector transfection. (e-j) RT-qPCR was conducted to measure the expressions of SCX, Mkx, COL1a1, Fmod, Mmp3 and Thbs4 after miR-378a-3p mimic and MAPK1 vector transfection. *P < 0.05, **P < 0.01, ***P < 0.001.

### Overexpression of MALAT1 repaired the damaged tendon tissues in rats

Finally, we established a rat tendon injury model to explore the function of MALAT1 *in vivo*. Compared with the CON group, the expression of MALAT1 dramatically decreased in the Model group and oe-MALAT1 group showed significantly increased MALAT1 expression (Figure 8(a)). In addition, compared with the CON group, the number of cells in the wound region increased in the Model group. The wound region in oe-MALAT1 group exhibited decreased cell numbers (Figure 8(b)). In addition, collagen type 1 and Thbs4 levels were lower in the Model group compared with the CON group, but higher in the oe-MALAT1 group compared with the Model group (Figure 8(c-d)).

The article "LncRNA MALAT1 promotes tenogenic differentiation of tendon-derived stem cells via regulating the miR-378a-3p/MAPK1 axis" was retracted in 2026. Reasons: concerns about the data; concerns about the results or conclusions.

**Figure 8.** Overexpression of MALAT1 relieve the impaired tendon tissues in the rats. (a) RT-qPCR were conducted to measure the MALAT1 expression. (b) HE staining of the tendon defect in the rats. (c-d) immunohistochemistry staining (Collagen type 1 and Thbs4) of tendon defect in the rats. *P < 0.05, **P < 0.01.

## Discussion

To date, there have been very few studies on the role of lncRNAs in the regulation of tenogenic differentiation, and the effects of MALAT1 on tenogenic differentiation have not been reported yet. To our knowledge, this study is the first to explore the role of MALAT1. In the current study, we confirmed that MALAT1 acts as a mediator of tenogenic differentiation and repair by regulating the miR-378a-3p/MAPK1 axis.

The role of lncRNA-mediated epigenetic regulation of transcription in various biological processes has attracted increasing attention [27]. MALAT1 was first discovered as an imprinted gene in non-small cell lung cancer [11]. Previous studies have shown that MALAT1 can specifically recruit members of the SR protein family, and participate in epigenetic and cell cycle regulation [28]. MALAT1 is highly expressed in a variety of tumors and can promote the proliferation, metastasis, and invasion of tumor cells [29,30]. In addition, MALAT1 also plays an important role in angiogenesis [31]. However, the effects of MALAT1 on tenogenic differentiation have not yet been reported. TDSCs are an ideal cell model for studying tendinopathy because of their self-renewal and differentiation abilities [32]. TGF-β1 has been confirmed to be an effective tenogenic inducer that stimulates the expression of tendon related transcription factors and marker genes, such as SCX, Mkx, COL1a1, Fmod, Mmp3, and Thbs4 [33,34]. In this study, we found that MALAT1 is upregulated in TGF-β1-treated TDSCs, and that SCX, Mkx, COL1a1, Fmod, Mmp3, and Thbs4 are downregulated after MALAT1 knockdown. These results indicate that MALAT1 plays an important role in tenogenic differentiation.

Recently, a growing number of studies have demonstrated that lncRNAs regulate various cellular biological activities as competing endogenous (ce) RNA or miRNA sponges. MALAT1 has been shown to be an miRNA sponge for miR-15b-5p in coronary atherosclerotic heart disease [35]. In lung cancer, MALAT1 acts as a ceRNA blocking miR-200a [30]. In addition, MALAT1 regulates the p38 MAPK/NF-κB signaling pathway by interacting with miR-125b, causing worsening of sepsis, heart inflammation, and dysfunction [36]. These findings indicate a negative correlation between MALAT1 and its target miRNAs. In this study, we found that MALAT1 was negatively regulated by miR-378a-3p in TDSCs. Knockdown of miR-378a-3p reversed the effects of si-MALAT1 on the tenogenic differentiation of TDSCs. These results revealed a novel role of MALAT1 in tendon injury. Studies have indicated that mitogen-activated protein kinase 1 (MAPK1) is a target gene for several miRNAs. Zhu et al. [35] found that MALAT1 suppresses autophagy and apoptosis in endothelial progenitor cells, and promotes cell viability via the miR-15b-5p/MAPK1 axis. Furthermore, MAPK1 was found to be negatively regulated by miRNA-127-5p [37], miR-490-3p [38], miRNA-433-5p [39] and other molecules. However, no studies so far have focused on the role of MAPK1 in tenogenic differentiation. Dual-luciferase reporter assay in this study indicated that MAPK1 shares complementary binding sites with miR-378a-3p. And overexpression of MAPK1 reversed the effects of miR-378a-3p mimic on the tenogenic differentiation of TDSCs. These results indicated that miR-378a-3p inhibits tenogenic differentiation by targeting MAPK1 expression.

The article "LncRNA MALAT1 promotes tenogenic differentiation of tendon-derived stem cells via regulating the miR-378a-3p/MAPK1 axis" was retracted in 2026. Reasons: concerns about the data; concerns about the results or conclusions.

Animal experiments are vital for the further study of lncRNAs in tendon injury. Therefore, in this study, we conducted animal experiments involving tendon injury in rats to further explore the role of MALAT1 in tenogenic differentiation. Consistent with the results of experiments on TDSCs, MALAT1 expression was downregulated in tendinopathy rats. Overexpression of MAPK1 significantly increased collagen type 1 and Thbs4 levels and decreased the number of cells in the wound region of tendinopathy rats. As a result, MALAT1 healed the damaged tendon tissues in rats.

## Conclusion

In summary, this study demonstrated that MALAT1 heals tendon injuries by inducing the tenogenic differentiation of TDSCs. Exploiting the MALAT1/miR-378a-3p/MAPK1 axis may therefore be a promising avenue for tendon injury treatment.

## Data Availability

The datasets used and analyzed during the current study are available from the corresponding author on reasonable request.
